# miR-124-3p Delivered Using Exosomes Attenuates the Keratinocyte Response to IL-17A Stimulation in Psoriasis

This article has been retracted.

**DOI:** 10.1155/2022/6264474

**Published:** 2022-10-12

**Authors:** Simin Liu, Jian Gong

**Affiliations:** ^1^School of Clinical Medicine, Jiangxi University of Chinese Medicine, Nanchang, Jiangxi 330004, China; ^2^Department of Integrated Traditional Chinese and Western Medicine, Dermatology Hospital of Jiangxi, Nanchang, Jiangxi 330001, China; ^3^Jiangxi Provincial Clinical Research Center for Skin Diseases, Nanchang, Jiangxi 330001, China

## Abstract

**Methods:**

NHEKs, HaCaT cells, and HEK 293T cells were treated with IL-17A. CCK-8 assays were performed to detect cell activity, and immunofluorescence staining and Western blotting were performed to detect the protein expression of STAT3. After isolation of exosomes via ultracentrifugation, the contents of miR-124-3p and oxidative stress markers such as superoxide dismutase (SOD), malondialdehyde (MDA), and glutathione peroxidase (GSH-Px) in keratinocytes were measured. Subsequently, transcriptomic analysis was performed using RNA-seq. Data were analysed by using the “edgeR” package within R. After verifying the abnormally expressed genes stimulated by IL-17A, a dual luciferase reporter assay was used to determine the interaction between miR-124-3p and STAT3. Finally, BALB/c mice were used to establish a psoriasis model for analysis. The effect of elevated miR-124-3p on the psoriasis mouse model was determined by exosomal delivery of miR-124-3p.

**Results:**

IL-17 intervention enhanced the cell activity of keratinocytes (*P* < 0.05). miR-124-3p was identified by RNA-seq as one of the differentially expressed miRNAs stimulated by IL-17A. miR-124-3p overexpression induced decreased STAT3 and MDA levels, increased SOD and GSH-Px levels in keratinocytes, and alleviated emergency responses of sclerosis damage (*P* < 0.05). The dual luciferase reporter assay results confirmed that STAT3 was regulated by miR-124-3p in a targeted manner (*P* < 0.05). Finally, miR-124-3p delivered by exosomes effectively alleviated the pathological manifestations and oxidative stress responses of psoriatic mice.

**Conclusions:**

miR-124-3p regulates keratinocyte activity via STAT3 in response to IL-17A stimulation. The ectopic expression of miR-124-3p in psoriatic skin reduces IL-17A-induced inflammation and inhibits the STAT3 pathway, thus alleviating the symptoms of psoriasis. The findings of this study suggest that exosomes can be used to therapeutically deliver miR-124-3p to keratinocytes and psoriatic lesions, which may provide novel insight for psoriasis treatment.

## 1. Introduction

Psoriasis is a common chronic papulosquamous skin disease characterized by sharply demarcated, erythematous, pruritic plaques with silvery scales. Plaques are commonly located in the trunk, limb extensor surfaces, and scalp [1]. Psoriasis occurs worldwide and presents in all ages, affecting 2–3% of people globally [2, 3] There are multiple types of psoriasis, including plaque psoriasis, which accounts for approximately 85% of cases, and pustular, guttate, palmoplantar, erythrodermic, and inverse psoriasis [4]. The infiltrating leukocytes in psoriasis patients release growth factors, cytokines, and chemokines such as VEGF, TNF-*α*, IL-17, IL-22, CXCL8, and CXCL2, affecting the proliferation and differentiation of epidermal keratinocytes, thus leading to the onset of disease. Recent studies have revealed that psoriasis is comorbid with multiple diseases, such as stroke, cardiometabolic disorder, and chronic kidney disease, resulting in overall reduced life expectancy and quality of life in patients [5]. Therefore, it is imperative to explore novel therapeutic strategies to improve the treatment of psoriasis.

Exosomes are nanosized vesicles (50-150 nm in diameter) released by various cells and play critical roles in intercellular communication in diverse biological and pathological processes [6]. There are proteins, mRNAs, and miRNA species within the exosomes. MicroRNAs (miRNAs) are small single-stranded noncoding RNAs of approximately 22 nucleotides that regulate gene expression posttranscriptionally by binding to target mRNAs [7]. miRNAs usually interact with the mRNA 3′UTR and, in some circumstances, with the CDS or 5′UTR to induce mRNA degradation and translational repression [8]. Previous studies have revealed that miRNAs regulate many biological functions, including inflammatory signalling pathways and DNA repair. Dysregulation of miRNAs is associated with multiple diseases, such as cancers, immune diseases, and psoriasis [9–12]. In recent studies, several miRNAs, such as miR-155, miR-378a, and miR-125, have been identified as dysregulated in psoriasis. miRNAs can be used as molecular therapeutics in the treatment of various diseases, and exosomes are currently an ideal vehicle for the delivery of miRNAs to diseased cells and tissues [13]. The significant effects of exosome-delivered miRNAs in recipient cells provide insight into psoriasis treatment [14].

Signal transducer and activator of transcription 3 (STAT3) is a transcription factor encoded by the STAT3 gene. STAT3 is involved in skin lesions of psoriasis. Previous studies have demonstrated that in skin lesions of psoriatic patients, STAT3 phosphorylation levels were higher than those in normal skin [15]*. In vivo* studies with transgenic mice demonstrated that constitutive activation of STAT3 in keratinocytes leads to skin lesions such as human psoriatic plaques [16]. STAT3 is essential for the differentiation of TH17 helper T cells, which contributes to many autoimmune diseases [17]. STAT3 also regulates the expression of genes that control cell survival, cell proliferation, and angiogenesis along with transcription factors such as NK-kB [18]. IL-6 and IL-20 family members, as well as some other cytokines and growth factors, can stimulate cells through activation of STAT3 [17]. In psoriasis, it has been shown that the IL-17, IL-22, and IL-23 signalling pathways are associated with STAT3. STAT3 has been validated as a promising therapeutic target in treating psoriasis [19, 20].

In this study, we aimed to investigate miRNAs that are associated with the pathogenesis of psoriasis. We conducted RNA sequencing to reveal dysregulated miRNAs within keratinocytes stimulated with IL-17 and successfully identified a panel of miRNAs differentially expressed in IL-17A-stimulated keratinocytes compared with nonstimulated controls. One of those miRNAs overexpressed in IL-17A-treated keratinocytes was miR-124-3p. We aimed to explore the function of miR-124-3p in vitro by overexpressing it in keratinocytes as well as *in vivo* by exosome delivery. We hypothesized that exosome-delivered miR-124-3p would alleviate psoriasis progression by targeting STAT3. Overall, our work validated the regulatory roles of miR-124-3p in response to cytokines in the context of psoriasis both *in vitro* and *in vivo*. The findings of our study may provide evidence for the application of exosome-delivered miRNAs in the treatment of autoimmune skin diseases.

## 2. Materials and Methods

### 2.1. Cell Culture and Cell Transfection

Normal human epidermal keratinocyte NHEKs (Cat. No. PCS-200-011) and human embryonic kidney cell lines HEK 293T cells (Cat. No. CRL-11268) were provided by the American Type Culture Collection (ATCC, Manassas, Virginia, USA). The human epidermal keratinocyte cell line HaCaT (Cat. No. GDC0106) was purchased from the China Center for Type Culture Collection (Wuhan, China). The cells were cultured in Dulbecco's modified Eagle's medium (DMEM) (Keygentec) in 5% CO_2_ at 37°C with 10% foetal bovine serum (Wisent) and 100 U/ml penicillin and streptomycin (Keygentec). For IL-17A treatment, HEK 293T cells or HaCaT cells were first seeded in 96-well plates at 1 × 104 cells/well and then starved overnight. The next day, IL-17A (R&D) was added to a final concentration of 100 ng/ml for the indicated times [21].

For cell transfection, miRNA mimics and a scrambled RNA fragment (negative control) were provided by RIBOBIO (Guangzhou, China). The cells were cultured in 6-well plates for 12 hr to reach 75% confluence. Then, 100 nmol/l miRNA mimics were transfected into cells using Lipofectamine according to the manufacturer's instructions (Thermo Fisher Scientific). Forty-eight hours after transfection, the cells were harvested and collected for subsequent assays.

### 2.2. CCK-8 Assay

After the indicated treatments, HaCaT cells were plated into 96-well plates at 1 × 104 cells per well. Twenty-four hours after transfection, the medium was replaced, and the cells were incubated with IL-17A (100 ng/ml) for up to 72 hrs. Next, 10 *μ*l of CCK-8 (Vazyme, Nanjing, China) reagent was added to each well at the indicated time points (0, 24, 48, and 72 h) and cultured for another 2 hr according to the manufacturer's instructions. The absorbance value was measured at 460 nm using a microplate reader (Bio-Rad, Hercules, CA, USA) [22].

### 2.3. Immunofluorescent Staining

HaCaT cells (1 × 104) were first plated on sterile cover slips in a 12-well plate. The next day, the cells were stimulated with the respective reagents (IL-17A, PeproTech, 100 ng/ml). After treatment, the cells were washed with PBS, fixed with 4% paraformaldehyde for 10 minutes, and then permeabilized with 0.1% Triton X-100 (Thermo Fisher Scientific) for 10 minutes. Following permeabilization, the cells were blocked with 2% bovine serum albumin for 1 hr and then incubated with primary antibodies overnight at 4°C (phospho-STAT3 Ab, AF3293, Affinity Biosciences; STAT3 Ab, AF6294, Affinity Biosciences). Next, the cells were incubated with dye-labelled secondary antibody for 1 hr at 37°C. Then, the cells were washed with PBS and incubated with FITC-labelled phalloidin (Thermo Fisher Scientific) for 30 minutes at room temperature. Images were captured by a confocal laser scanning microscope (FV3000, Olympus, Japan) and analysed using ImageJ software [23].

### 2.4. RT–qPCR

First, samples were isolated with TRIzol reagent (Invitrogen), and total RNA was extracted following chloroform extraction and isopropanol precipitation. cDNA synthesis was performed with a HiScript II One Step RT–PCR Kit (Vazyme). Real-time PCR was performed with ChamQ Universal SYBR qPCR Master Mix (Vazyme). The expression level of genes was normalized to GAPDH and analysed by the 2^−*ΔΔ*Ct^ method. For miRNA quantification, total RNA was first reverse transcribed with a miRNA reverse transcription kit (Thermo Fisher Scientific), including primers for miR-124-3p (Thermo Fisher Scientific). The relative level of miR-124-3p was normalized to U6 using the 2^−*ΔΔ*Ct^ method [24].

### 2.5. Exosome Isolation and Quantification

Exosomes were isolated with the ultracentrifugation method following a publicly available protocol [25]. Briefly, first, the cell supernatant containing exosomes was centrifuged at approximately 300 × g for 5 minutes to remove cells and then centrifuged at 12,000 × g for 45 minutes to remove debris. Next, the supernatant was collected and filtered through 0.22 *μ*m filters (Merck Millipore) to remove microvesicles, cell debris, and other large particles. Finally, the filtered supernatant was centrifuged in a Beckman Coulter Ultracentrifuge at 100,000 × g at 4°C for 90 minutes to obtain pellet exosomes. After washing with PBS and centrifuging at 120,000 × g for 90 minutes, the purified exosomes were quantified with a Human Exosome ELISA Kit (Novus) according to the manufacturer's instructions.

### 2.6. Exosome Characterization with Nanoparticle Tracking Analysis

Purified exosomes (100 *μ*l) were analysed with a NanoSight LM10-HSB instrument (A&P Instrument Co.) for nanoparticle tracking analysis (NTA) at room temperature. The mean size of exosomes and size distribution data were analysed with NTA 2.2 software [25].

### 2.7. Loading miR-124-3p into Exosomes with Electroporation

To load miR-24-3p into the exosomes, 50 *μ*g miR-124-3p mimic was gently mixed with 100 *μ*g purified exosomes in 200 *μ*l electroporation buffer at 4°C [25]. After electroporation at 400 V and 50 *μ*F for three cycles with a 30 ms pulse/2 s pause, the mixture was incubated at 37°C for 30 min and centrifuged at 100,000 × g for 70 min to remove unbound miR-24-3p. Exosomes were then isolated as described above and washed once with cold PBS. RNA was extracted from pellets using TRIzol reagent (Invitrogen), and the loading efficiency of miR-124-3p into exosomes was measured with RT–qPCR.

### 2.8. Western Blot

To prepare whole-cell lysates, samples were first lysed with RIPA buffer (Beyotime, Shanghai, China) on ice and then centrifuged at 13,000 × g for 10 minutes at 4°C. The protein concentration was measured using a bicinchoninic acid (BCA) protein assay kit (CWBIO). An equal amount of protein was separated by 12% SDS–PAGE. Following separation through electrophoresis, the proteins were transferred to PVDF membranes. After blocking with 5% nonfat milk or 2% BSA, the membrane was incubated with primary antibodies at 4°C overnight (phospho-STAT3 Ab, AF3293, Affinity Biosciences; STAT3 Ab AF6294, Affinity Biosciences) with actin as a loading control and then incubated at room temperature with HRP-conjugated secondary antibodies for 1 hr in the dark. The signal was developed with ECL Reagent (Beyotime) according to the manufacturer's directions and imaged with a chemiluminescent imaging system ChemiDoc (Bio-Rad) [26].

### 2.9. Transcriptomic Analysis and Enrichment Analysis

Transcriptomic analysis was performed using RNA-seq. Data were analysed by using the “edgeR” package within R [27]. Enrichment analysis was performed with the “clusterProfiler” package within R [28].

### 2.10. Dual-Luciferase Reporter Assay

#### 2.10.1. Plasmid Construction

The target sequences of miR-124-3p in STAT3 were predicted by the StarmirDB database (https://sfold.wadsworth.org/starmirDB.php). Wild-type STAT3 3′UTR sequences containing the miR-124-3p binding sites were amplified by PCR, and mutant sequences were constructed by site-directed mutagenesis by substituting the seed regions with miR-124-3p. The wild-type or mutant STAT3 plasmids were synthesized and constructed by GenScript (Nanjing, China) and inserted into the pmirGLO plasmid (GenePharma). HEK 293T cells were seeded in 24-well plates at 1 × 104 cells/well and cultured to 80% confluence before transfection. Subsequently, luciferase constructs were cotransfected with miR-124-3p mimic or scramble miRNAs into HEK 293T cells using Lipofectamine 3000 following the manufacturer's manual. The Dual-Luciferase Reporter Assay System (Promega) was used to measure the luciferase activity after incubation for 48 hr.

#### 2.10.2. Mouse Model

Wild-type male BALB/c mice (8 weeks, 20-25 g) were purchased from Beijing Vital River Laboratory Animal Technology. To overexpress miR-124-3p, 3 *μ*g human miR-124-3p mimic or scramble miRNA mimics were packaged in Invivofectamine 3.0 Reagent or 50 *μ*g exosomes containing miR-124-3p were injected into the shaved back skin of BALB/c mice at Days 0, 1, and 3 intradermally [29]. To establish psoriasis mouse models, the backs of the mice were shaved with a 2 × 3 cm area, and 50 mg 5% imiquimod (IMQ, MedChemExpress) was applied topically to this area [30]. Vernier callipers (Deli) were used to measure the back skin thickness every 2 days at three different sites within IMQ-treated regions. Scales 0 to 4 (0, healthy; 1, mild; 2, moderate; 3, severe; and 4, very severe) were assigned by three independent researchers for erythema, scaling, and thickness of the IMQ-treated region. The Ethics Committee for Animal Research of School of Clinical Medicine, Jiangxi University of Chinese Medicine, reviewed and approved the experimental protocols.

#### 2.10.3. Histopathology and Immunohistochemistry Staining

The mouse skin tissues were excised, washed with PBS, fixed in formalin, embedded in paraffin, and sliced into 5 *μ*m sections. Then, the tissue sections were stained with haematoxylin for 10 minutes and eosin (Sigma–Aldrich) for 3 minutes at room temperature and observed under a light microscope (Olympus) for histological evaluation. For immunohistochemistry staining, the slides were first deparaffinized. Antigen retrieval was performed at 100°C for 20 minutes in a steamer in 0.01 M sodium citrate buffer with pH 6.0. After blocking with 1% BSA for 30 min at room temperature, the cells were incubated with primary antibody (Ki67 Ab, AF0198, Affinity Biosciences; phospho-STAT3 Ab, AF3293, Affinity Biosciences; STAT3 Ab, AF6294, Affinity Biosciences) for 45 min and HRP-conjugated secondary antibody for 30 min at room temperature. A DAB Horseradish Peroxidase Colour Development Kit (Beyotime) was applied, and the sections were incubated for approximately 3 minutes. The images were observed and photographed using a light microscope [30].

#### 2.10.4. Statistical Analysis

Statistical analysis was performed with R. Data are presented as the mean ± standard deviation (SD). Differences between groups were evaluated by a *t-*test or one-way analysis of variance (ANOVA). A *p* value less than 0.05 was regarded as statistically significant.

## 3. Results

In this study, we explored the function and regulatory mechanism of miR-124-3p in psoriasis progression *in vitro* and *in vivo*. miR-124-3p was downregulated in IL-17A-treated keratinocytes as well as in skin samples from psoriasis patients. STAT3 was directly targeted by miR-124-3p, and miR-124-3p overexpression reversed the IL-17A-induced increase in STAT3 expression in keratinocytes. miR-124-3p overexpression inhibited IL-17-enhanced proliferation, reduced oxidative stress in keratinocytes *in vitro*, and attenuated inflammation and skin thickness in psoriasis mouse models. The findings of our study may provide potential therapeutic targets for psoriasis treatment.

### 3.1. miR-124-3p Inhibits IL-17A-Mediated Keratinocyte Proliferation

We identified 67 miRNAs differentially expressed at least 2-fold in NHEKs stimulated with IL-17 and 57 miRNAs differentially expressed at least 2-fold in HaCaT cells stimulated with IL-17 (Figures 1(a) and 1(b)). Among them, 5 miRNAs were upregulated in both cell lines (Figure 1(c)), and 7 miRNAs were downregulated in both cell lines (Figure 1(c)), and they were further confirmed in patient samples in the public dataset GSE174763. miR-124-3p was significantly downregulated in IL-17A-stimulated keratinocytes, as well as in keratinocytes from psoriatic skin lesions (Figure 1(d)). The results of RT–qPCR analysis confirmed the decreased levels of miR-124-3p in keratinocytes treated with IL-17A (Figure 1(e)). We next tested whether miR-124-3p had functional roles in keratinocytes. We stimulated cells with IL-17A and found that IL-17A increased cell proliferation, while overexpression of miR-124-3p in HaCaT cells reduced the proliferation rate induced by IL-17A (Figure 1(f)).

### 3.2. miR-124-3p Inhibits STAT3 in Keratinocytes

As dysregulation of miRNAs in psoriatic keratinocytes may affect the pathogenesis of psoriasis, we explored the potential role of miR-124-3p. We overexpressed miR-124-3p in keratinocytes and performed RNA-seq. As shown in Figure 2(a), 117 genes were upregulated at least 2-fold, and 208 genes were downregulated at least 2-fold. By intersecting the genes with miR-124-3p predicted targets, we found that STAT3 was a potential gene directly targeted by miR-124-3p (Figure 2(b)). When we overexpressed miR-124-3p in keratinocytes in vitro, we found that STAT3 mRNA levels decreased (Figure 2(c)) as well as the protein level (Figure 2(d)). We then stimulated HaCaT cells with IL-17 and found that STAT3 expression levels increased. Overexpression of miR-124-3p reduced the STAT3 level as well as p-STAT3 level even in the presence of IL-17 stimulation (Figures 2(e) and 2(f)).

### 3.3. miR-124-3p Affects Oxidative Stress Responses in Keratinocytes

To confirm the influence of miR-124-3p on oxidative stress in keratinocytes, we measured the oxidative stress markers SOD, MDA, and GSH-Px in cells. The results also showed increased SOD and GSH-Px and decreased MDA at the mRNA level when miR-124-3p was overexpressed in keratinocytes in vitro, which was completely contrary to the results after IL-17 stimulation (decreased SOD and GSH-Px mRNA and elevated MDA mRNA after IL-17 stimulation) (Figures 3(a)–3(c)).

### 3.4. miR-124-3p Directly Targeted STAT3 in Keratinocytes

To test whether miR-124-3p directly targets STAT3, we performed luciferase reporter assays. As shown in Figure 4(a), the StarmirDB database (https://sfold.wadsworth.org/starmirDB.php) predicted multiple miR-124-3p binding sites in the STAT3 mRNA 3'UTR. We cloned miR-124-3p binding sites as well as mutant sequences in luciferase constructs (Figure 4(b)). As shown in Figure 4(c), overexpression of miR-124-3p reduced luciferase activity compared to scramble miRNAs in site 1, site 2, site 4, CDS segment, and 3′UTR segment constructs, while the luciferase activity was partially recovered in seed region mutant constructs. When we cotransfected miR-124-3p and the 3′UTR segment in HaCaT cells, we found that the STAT3 expression level was higher than that in cells transfected with only miR-124-3p (Figure 4(d)). These results indicated that miR-124-3p directly targets the STAT3 3′UTR, thus regulating protein expression.

### 3.5. In Vitro Delivery of miR-124-3p in HaCaT Cells with Exosomes as Delivery Cargo

Previous studies have shown that exosomes can be used as cargo to deliver miRNAs or siRNAs; thus, we tested whether miR-124-3p can be delivered via engineered exosomes. We used 2 different methods to generate exosomes containing miR-124-3p as described in previous studies [25, 31]. In the first method, we stably expressed miR-124-3p in HEK 293T cells and purified exosomes after 48 hr of incubation. In the second method, we first purified exosomes from regular HEK 293T cells and loaded miR-124-3p mimics using electroporation. As shown in Figure 5(a), both methods resulted in exosomes loaded with miR-124-3p, with electroporation demonstrating higher yield but larger variation. When we incubated the exosomes with HaCaT cells, we found that exosomes generated by both methods had similar efficiency in fusion with HaCaT cells and delivered miR-124-3p into cells, as shown in Figure 5(b). When HaCaT cells were stimulated with IL-17A, we found that incubation with exosomes containing miR-124-3p reduced STAT3 expression in the presence of IL-17A stimulation (Figures 5(c), 5(f), and 5(g)) and reduced the cell proliferation rate induced by IL-17A (Figure 5(d)). qPCR analysis of psoriasis-related genes showed that CXCR5, IL22, KRT16, IL17C, CXCL1, and CCL20 expression was also reduced in cells incubated with exosomes containing miR-124-3p, which was similar to the effect of transfection with miR-124-3p mimic by RNAiMAX (Figure 5(e)).

### 3.6. *In Vivo* Delivery of miR-124-3p with Exosomes Reduced IMQ-Induced Psoriasis

Then, we tried to determine whether *in vivo* delivery of miR-124-3p could relieve IMQ-induced psoriasis in BALB/c mice. Synthetic miR-124-3p mimics or exosomes containing miR-124-3p were injected into the back skin of mice treated with IMQ (Figure 6(a)). As expected, IMQ treatment caused erythema and induced cell proliferation (Figure 6(b)). The skin thickness also increased after IMQ treatment. Intradermal delivery of miR-124-3p by exosomes increased miR-124-3p levels in mouse skin (Figure 6(d)). Clinical scores showed that miR-124-3p overexpression relieved skin inflammation and reduced skin thickness (Figure 6(c)). Delivery of miR-124-3p with Invivofectamine also relieved the symptoms caused by IMQ. In histological analysis, we found that the epidermal thickness significantly decreased in the miR-124-3p-treated groups. Ki67 staining within skin samples showed that the number of proliferating cells decreased in mice injected with miR-124-3p (Figure 6(b)). In addition, qPCR showed that some psoriasis-related genes, such as Ccl20, Cxcr5, Krt16, and Il17c, significantly decreased when miR-124-3p was overexpressed *in vivo*. (Figure 6(e)). Finally, analysis of oxidative stress markers also revealed that when miR-124-3p was overexpressed in mice, SOD and GSH-Px increased, while MDA decreased, suggesting effectively controlled oxidative stress responses (Figure 6(f)). Taken together, our results showed that increased miR-124-3p expression could reduce psoriasis-like skin inflammation, and delivery of miR-124-3p could be a potential therapy to treat psoriasis *in vivo*.

## 4. Discussion

In this study, we found that miR-124-3p attenuated the inflammatory responses caused by IL-17A in keratinocytes. The expression of miR-124-3p was decreased in IL-17A-treated keratinocytes. miR-124-3p overexpression reversed the increase in STAT3 expression and keratinocyte proliferation rate induced by IL-17A treatment. The oxidative stress and expression of psoriasis-related genes were inhibited by the delivery of exosomes carrying miR-124-3p *in vivo*. Our findings suggest miR-124-3p as a potential therapeutic target for psoriasis treatment.

Recent studies have shown that keratinocytes play important roles in modulating skin inflammation instead of acting as passive targets within the skin immunity environment [32]. Knockout of IL-17RA in keratinocytes in mice attenuated skin inflammation caused by IMQ, while IL-17RA knockout in other cell types did not show attenuation, indicating that keratinocytes are key targeting cells for IL-17A-induced psoriasis [33]. In our study, we found that IL-17A treatment significantly enhanced the proliferation potential of keratinocytes, which was consistent with previous findings. miR-124-3p directly targeted STAT3 in keratinocytes. STAT3 plays critical roles in regulating inflammatory responses and is important for epidermal homeostasis within skin. STAT3 is activated in keratinocytes of psoriatic lesions and promotes the proliferation of keratinocytes. Previous studies have shown that the topical application of a STAT3 inhibitor could inhibit psoriasis onset in a mouse model [19] and in clinical trials [20]. In this study, we found that the expression of STAT3 was negatively regulated by miR-124-3p in psoriasis, and STAT3 expression showed a significant increase after stimulation with IL-17A, which was consistent with previous studies. In addition, the oxidative stress reaction is an important pathological process in the development of psoriasis. Keratinocytes stimulated by inflammatory reactions can cause serious inflammatory changes and destroy the original functions of cells. A study also indicated that oxidative stress caused by reactive oxygen species also promotes psoriasis by activating STAT3 [34]. We have found in previous studies that the peripheral blood of psoriasis patients is clearly hyperoxidized [35], which is consistent with our research (after IL-17 stimulation, SOD and GSH-Px in cells decreased, but MDA increased), further supporting the relationship between psoriasis and oxidative stress injury. Moreover, significant alleviation of oxidative stress responses was observed in keratinocytes and psoriatic mice after miR-124-3p was elevated, while miR-124-3p inhibition exhibited the opposite effects on oxidative stress in keratinocytes. The results of *in vivo* assays demonstrated that STAT3 was highly expressed in the skin lesions of psoriatic rats, and miR-124-3p, which directly targets STAT3 at the 3′UTR, reduced the severity of psoriatic lesions induced by IMQ in mice, which was consistent with previous findings. These results indicate that STAT3 could be an effective therapeutic target in psoriasis treatment.

Although liposomes such as Invivofectamine used in this study could effectively deliver miRNAs *in vivo*, this reagent is not suitable for use in clinical practice due to stability, safety, and off-target effects [36, 37]. A previous study showed that exosomes purified from cells transfected with let-7a miRNA could inhibit cancer cell growth in mice [38]. These results indicate that exosomes are a promising cargo in clinical practice for DNA or RNA delivery with multiple advantages over liposomes. In our study, we revealed that HEK 293T cells stably transfected with miR-124-3p could generate exosomes containing abundant miR-124-3p. Compared to electroporation, this method is more convenient and avoids the problem of aggregation seen in electroporation. The different cells and miRNA mimics used compared with previous studies may cause the difference in miRNA introduction efficiency. Furthermore, we compared the effect of the exosome delivery system *in vitro* and found that exosomes containing miR-124-3p stably overexpressing miR-124-3p constructs in HEK 293 T cells were more efficient than electroporation. Moreover, compared to delivering miR-124-3p with Invivofectamine *in vivo*, exosomes were safer and exhibited fewer side effects in mice injected with exosomes. Our findings may provide novel insight into antipsoriasis therapy.

However, there are still some limitations in this study. First, the mechanism of exosome-mediated communication between HEK 293T and HaCaT cells was not explored. Second, whether STAT3 overexpression could rescue the effects of miR-124-3p delivered by exosomes remains to be further investigated. Third, the clinical application of engineered exosomes is challenged by the comprehensive molecular and functional characterization before each treatment, which requires the improvement of automatic preparation of disease-targeted exosomes in the future.

## 5. Conclusion

miR-124-3p modulates keratinocyte activity via STAT3 upon stimulation by IL-17A. Ectopic expression of miR-124-3p in psoriatic skin alleviates IL-17A-induced inflammation and inhibits the STAT3 pathway, thus relieving psoriatic symptoms.

## Figures and Tables

**Figure 1:** miR-124-3p inhibits IL-17A-mediated keratinocyte proliferation. RNA extracted from NHEKs treated with IL-17 (*n* = 3), HaCaT cells treated with IL-17A (*n* = 3), and PBS-treated control cells (*n* = 3) was used for small RNA-seq. (a) Venn diagrams showing 6 upregulated microRNAs in both NHEKs and HaCaT cells treated with IL-17A. (b) Venn diagrams showed 12 downregulated microRNAs in both NHEKs and HaCaT cells treated with IL-17A. (c) Venn diagrams showed that 5 upregulated microRNAs were also upregulated in lesioned skin samples in the GSE174763 dataset. (d) Venn diagrams showed that 7 downregulated microRNAs were also downregulated in lesioned skin samples in the GSE174763 dataset. (e) qPCR analysis of miR-124-3p in HaCaT cells treated with IL-17A (*n* = 6) and PBS (*n* = 6). The expression level was normalized to U6. (f) CCK-8 assay of cells treated with IL-17A and miR-124-3p at 0, 24, 48, and 72 hrs. ^∗^*p* < 0.05,  ^∗∗^*p* < 0.01, and^∗∗∗^*p* < 0.001.

**Figure 2:** miR-124-3p inhibits STAT3 in keratinocytes. RNA extracted from HaCaT cells transfected with miR-124-3p (*n* = 3) and scramble miRNA (*n* = 3) was used for RNA-seq. (a) A total of 208 genes were downregulated, and 117 genes were upregulated in HaCaT cells transfected with miR-124-3p. (b) Transcript count of STAT3 in sequencing samples from cells treated with scramble miRNAs or miR-124-3p mimic. (c) qPCR analysis of STAT3 expression in HaCaT cells transfected with miR-124-3p mimic or miR-124-3p inhibitor. Data were normalized to GAPDH. (d) Western blot analysis of STAT3 and p-STAT3 protein expression in HaCaT cells transfected with miR-124-3p mimic or miR-124-3p inhibitor. Actin was used as a loading control. (e) Immunostaining of STAT3 in HaCaT cells treated with IL-17A and miR-124-3p. (f) Immunostaining of p-STAT3 in HaCaT cells treated with IL-17A and miR-124-3p. ^∗^*p* < 0.05,  ^∗∗^*p* < 0.01, and^∗∗∗^*p* < 0.001.

**Figure 3:** miR-124-3p affects oxidative stress responses in keratinocytes. (a) The mRNA levels of SOD in keratinocytes after the indicated treatments. (b) GSH-Px mRNA levels in keratinocytes after the indicated transfections. (c) MDA mRNA levels in keratinocytes after the indicated transfections. ^∗^*p* < 0.05,  ^∗∗^*p* < 0.01, and^∗∗∗^*p* < 0.001.

**Figure 4:** miR-124-3p directly targeted STAT3 in keratinocytes. (a) Graph showing the luciferase constructs used to confirm the direct targeting of STAT3 mRNA by miR-124-3p. (b) Graph showing the predicted binding sites of miR-124-3p in STAT3 mRNA and designed mutant sequences used in the luciferase assay. (c) Luciferase activity in HEK 293T cells cotransfected with the respective constructs and miR-124-3p mimic or scramble miRNAs. (d) Western blot analysis showed that cotransfection of the STAT3 3′UTR segment and miR-124-3p could rescue the miR-124-3p downregulating effect on STAT3 in HaCaT cells. ^∗^*p* < 0.05,  ^∗∗^*p* < 0.01, and^∗∗∗^*p* < 0.001;  ^#^*p* < 0.05,  ^##^*p* < 0.01, and^###^*p* < 0.001. ^∗^wild-type sequence vs. vector; ^#^mutant sequence vs. wild-type sequence.

**Figure 5:** *In vitro* delivery of miR-124-3p in HaCaT cells with exosomes as delivery cargo. (a) qPCR analysis of miR-124-3p levels in exosomes from the miR-124-3p overexpression stable cell line (Exosome_ov), electroporation-treated exosomes (Exosome_elec), and exosomes from the scramble miRNA overexpression stable cell line (Exosome_ev). The miR-124-3p mimic (Synthetic_mimic) was used as a positive control. (b) qPCR analysis of miR-124-3p levels in cells coincubated with Exosome_ev, Exosome_ov, and Exosome_elec. Cells transfected with scramble by RNAiMax were used as a negative control, and cells transfected with miR-124-3p mimic were used as a positive control. (c) Western blot showing STAT3 protein expression in HaCaT cells coincubated with Exosome_ov or Exosome_elec. (d) CCK-8 assay of cells treated with IL-17A and Exosome_ov, Exosome_elec, Exosome_ev, or miR-124-3p at 0, 24, 48, and 72 hrs. (e) qPCR analysis of CXCR5, IL22, KRT16, IL17C, CXCL1, and CCL20 expression in HaCaT cells treated with IL-17A and Exosome_ov, Exosome_elec, Exosome_ev, or miR-124-3p. (f) Immunostaining of STAT3 in HaCaT cells coincubated with Exosome_ov or Exosome_elec and IL-17A. (g) Immunostaining of p-STAT3 in HaCaT cells coincubated with Exosome_ov or Exosome_elec and IL-17A. ^∗^*p* < 0.05,  ^∗∗^*p* < 0.01, and^∗∗∗^*p* < 0.001.

**Figure 6:** *In vivo* delivery of miR-124-3p with exosomes reduced IMQ-induced psoriasis. (a) Graph showing the experimental design. (b) Graph showing the back skin of mice, H&E staining of back skin samples, and IHC staining for Ki67, STAT3, and p-STAT3 protein in back skin samples from mice injected with Exosome_ov, miR-124-3p or scramble miRNAs in combination with IMQ. (c) Clinical scores of mouse back skins in each group (*n* = 10). (d) qPCR analysis of miR-124-3p levels in the back skin samples of the corresponding mouse model (*n* = 5). (e) qPCR analysis of Cxcr5, Il22, Krt16, Il17c, Cxcl1 and Ccl20 expression in the back skin samples of the corresponding mouse model (*n* = 5). (f) The results of oxidative stress damage. ^∗^*p* < 0.05,  ^∗∗^*p* < 0.01, and^∗∗∗^*p* < 0.001.

## Data Availability

The datasets used and/or analysed during the current study are available from the corresponding author on reasonable request.
